# circFAT1(e2) Inhibits Cell Apoptosis and Facilitates Progression in Vascular Smooth Muscle Cells through miR-298/MYB Axis

**DOI:** 10.1155/2021/1922366

**Published:** 2021-12-13

**Authors:** Zhenhua Shi, Shiyong Ye, Yijia Xiang, Daying Wu, Jian Xu, Jianqiang Yu, Chunlai Zeng, Jun Jiang, Wuming Hu

**Affiliations:** ^1^Department of Cardiology, Lishui Municipal Central Hospital, 289 Kuocang Road, 323000 Lishui, Zhejiang, China; ^2^State Key Laboratory of Genetic Engineering, School of Life Sciences, Fudan University, Shanghai 200438, China

## Abstract

Presently, as one of the three types of muscles in the human body, smooth muscle carries out many biological activities. Meanwhile, its abnormal development also leads to many diseases. Circular RNA, belonging to the noncoding RNA family, is demonstrated to function importantly in various diseases including smooth muscle. Here, we assumed circFAT1(e2) probably exhibited a primary role in vascular smooth muscle. Therefore, we conducted cell viability and cell apoptosis assay to validate the effects of circFAT1(e2) on vascular smooth muscle progression. Then, we supposed miR-298 was one target of circFAT1(e2) and executed corresponding experiments to test this hypothesis. Dual-luciferase reporter assay indicated miR-298 could bind to circFAT1(e2) and then modulated MYB level, thus regulating smooth muscle progression. Subsequently, based on the GSE41177 dataset, we identified 1982 differentially expressed genes (DEGs) in atrial fibrillation, and all DEGs were upregulated, including MYB. Finally, enrichment analysis of upregulated genes indicated that they were related to endodermal cell differentiation. The protein-protein interaction network revealed that EGFR, GNG2, and FPR2 were related to atrial fibrillation. In conclusion, our data find that circFAT1(e2) sponges miR-298 and then regulates MYB expression, thus affecting atrial fibrillation progression. Our findings provide a newly produced indicator and target for vascular smooth muscle diagnosis and treatment.

## 1. Introduction

Smooth muscle is the nonstriated muscle tissue, is ubiquitous in the walls of human arteries and veins, has male and female reproductive tracts, and so on [1]. Although the functional traits of smooth muscle in multiple organs can be distinguished greatly, it can generally be divided into two categories: multiunit and single-unit smooth muscle [2]. The abnormal expressions of smooth muscle in different tissues can lead to leiomyoma, bronchial asthma, gallstones, kidney and ureteral stones, and so on [3]. Leiomyoma belongs to benign tumors of skin smooth muscle cells, caused by abnormal proliferation of smooth muscles [4]. The treatment of leiomyomas is mainly surgical resection. The tumor should be excised completely in case of high recurrence [5]. Therefore, the latent mechanism of smooth muscle is still vital to study.

MYB is a transcription factor that displays importance in regulating hematopoietic cell proliferation and differentiation. Its cellular counterpart is subsequently separated as c-MYB. It is highly increased in the thymus, hematopoietic cells, and nerve tissues and necessary for erythroid maturation and T and B lymphocyte development. It is worth noting that c-MYB is essential for human survival and deletion of two alleles of this gene in an embryonic stem cell can cause its death. Moreover, c-MYB also serves as a vital role in the generation of vascular smooth muscle cells (VSMCs) from embryonic stem cells (ESCs). ESCs give rise to progenitor cells that express vascular endothelial growth factor receptor type-2 (VEGFR-2) and then give rise to VSMCs in a process involving c-MYB. c-MYB not only activates the expression of VEGFR2 but also enables the ability of VEGFR2^+^ progenitor cells to differentiate into VSMCs.

In the last two decades, several proteomics studies have revealed dysregulation of multiple genes can support malignant transformation [6]. Circular RNA, a sort of naturally occurring noncoding RNA, is highly expressed in abnormally expressed smooth muscle [7]. Although the function and mechanism of circular RNA are not well understood, recent researches have revealed circRNA is probably considered as potential molecular indicators for the diagnosis and treatment of numerous diseases [8]. Up to date, some breaking researches are focusing on the links between circRNAs and cancers and finally arrive at solid conclusions. circRNA regulates gene expression by affecting the transcription, mRNA conversion, and translation of RNA binding proteins and microRNA [9]. Some circRNAs regulate the expression of messenger RNA (mRNA) by acting as a microRNA (miRNA) sponge. In lung cancer, hsa_circRNA_101237 promotes the expression of MAPK1 through miRNA-490-3p sponge, thereby affecting NSCLC as an important onco-circRNA [10]. In hepatocellular carcinoma, circRNA-5692 inhibits the progression of hepatocellular carcinoma by enhancing DAB2IP expression through sponge miR-328-5p [11]. However, no reports on the association between circRNA and smooth muscle are shown.

Presently, circRNA is identified to display importance in smooth muscle with next-generation sequencing methods emerging, like RNA sequencing [12]. circRNA hsa_circ_0132266 (circ_0132266) is abated in the peripheral blood mononuclear cells (PBMCs) of smooth muscle patients and can sponge miR-337-3p to suppress PML and then reduce cell viability [13]. circFAT1(e2) is overexpressed in smooth muscle cells and acts as a promoter to induce cell viability and cell cycle, but retard cell apoptosis, compared to normal cells [14]. Thus, it would be a promising field to study circRNA mechanisms in smooth muscle.

We here attempt to detect circFAT1(e2) functions in vascular smooth muscle. CCK-8 assay and cell apoptosis analysis are conducted to reveal the function of circFAT1(e2) in vascular smooth muscle. Our data reveal miR-298 interplay with circFAT1(e2) and then affect downstream target MYB expression. Then, we identify differential expression genes (DEGs) between patients with atrial fibrillation and normal people using dataset GSE41177. Finally, GO, KEGG, and PPI analyses are conducted to illustrate the potential mechanism of upregulated DEGs in atrial fibrillation.

## 2. Materials and Methods

### 2.1. Dataset and Differential Expression Genes

The gene expression dataset GSE41177 which included 16 left atria junctions of patients with atrial fibrillation and 3 controls was obtained in Gene Expression Omnibus (GEO, https://www.ncbi.nlm.nih.gov/geo/query/acc.cgi). GEO is an international open repository of storage and free-used microarrays, second-generation sequencing, and high-throughput functional genomic datasets with other forms. The limma package in R was employed for upregulated differential expression genes (DEGs) identification between patients with atrial fibrillation and normal people. The cut-off criteria were FC > 1.5 and *P* < 0.001; FC stands for fold change.

### 2.2. Enrichment Analysis of Kyoto Encyclopedia of Genes and Genomes (KEGG) Pathway and Gene Ontology (GO) Term

KEGG is a database for the comprehensive analysis of gene functions based on networks of genes and molecules. GO is a knowledgebase for annotating genes and their products from the aspects of biological process (BP), cell component (CC), and molecular function (MF). The Database for Annotation, Visualization and Integrated Discovery (DAVID) is a systematic online tool providing a systematic set of functional annotation information of genes and proteins, so that researchers can acquire biological information. KEGG pathway and GO term enrichment analysis were carried out using DAVID. *P* less than 0.05 was significant in statistics.

### 2.3. Protein-Protein Interaction (PPI) Network

PPI network reveals the interactions among protein molecules, which is vital to achieving a detailed description of their functions and relevant mechanisms in organisms. Presently, PPI is annotated at many online resources, including the Search Tool for the Retrieval of Interacting Genes/Proteins database (STRING, http://string-db.org/) which provides multiple perspectives. In this study, the PPI network of upregulated DEGs was constructed by STRING.

### 2.4. Cell Culture and Transfection

HUASMC and HASMC cells (human smooth muscle cell lines) got both ordered from the American Type Culture Collection. Both of them were incubated in DMEM (Invitrogen, USA) added with 10% FBS (Biochrom, USA) under a 37°C incubator with 10% CO_2_. The abovementioned cells were transfected with demonstrated plasmids by Lipofectamine 2000 (Invitrogen, USA) as the manual described. The sequence of siRNAs was as follows: si-circFAT1(e2): 5′-GAGACAGATTCCCGACAGTTA-3′ and si-NC: 5′-UUCUCCGAACGUGUCACGUTT-3′.

### 2.5. Cell Viability Assay

3 × 10^3^ VSMCs after sorting in each well were reseeded into 96-well plates as indicated. Cell proliferation assay was conducted on the following day. 10 *μ*l of CCK-8 solution (Dojin Laboratories, Kumamoto, Japan) was put down at scheduled times for 2 h incubation. Absorbance value in 450 nm was detected by a spectrophotometer. The representative data indicated cell viability.

### 2.6. Cell Apoptosis Assay

Cells were firstly fixed with 70% precold ethanol and then grew in RNase A. Then, VSMCs stained with Annexin V/PI reagent (eBioscience, USA) were subjected to FACS analysis for cell apoptosis measurement using flow cytometry (BD Biosciences, San Jose, CA, USA).

### 2.7. Reverse Transcription and qRT-PCR

TRIzol reagent (Invitrogen, USA) was prepared to extract total RNA from cells and tissues as the manual's description. Reverse transcription system was conducted as follows: 10 *μ*l volume included 500 ng RNA with PrimeScript RT Reagent Kit (Invitrogen, USA) and RNase-free ddH_2_O, followed by subjecting to qRT-PCR with SYBR Premix Ex Taq (TaKaRa, China). The pertinent RNA expression was measured by the 2^−*ΔΔ*Ct^ method. The primers were as follows: circFAT1(e2): forward 5′-AACAGAAGAGAACTGGGGCG-3′, reverse 5′-GATCAGGGTGCCAATGGTGA-3′; miR-298: forward 5′-GGCAGAGGAGGGC-3′, reverse 5′-GTGCGTGTCGTGGAGT-3′; MYB: forward 5′-ACATCTCCAGTCACGTTCCC-3′, reverse 5′-GGATCCTCACATGACCAGAGTTCGAG-3′; and GAPDH: forward 5′-TGTTCGTCATGGGTGTGAAC-3′, reverse 5′-ATGGCATGGACTGTGGTCAT-3′.

### 2.8. Luciferase Reporter Assay

The binding sites of miRNAs and circFAT1(e2) are predicted based on the web-based program CircInteractome [15]. The molecular targets of miR-298 are predicted using the online database starBase (based on miRNA target prediction programs, namely, TargetScan, miRanda, microT, PITA, miRmap, and PicTar) [16]. Wild-type (WT) or mutated circ-FAT1(e2) with the assumed binding site was amplified and then inserted into pmirGLO construct (Promega, USA). Similarly, WT or mutated sequence of MYB 3′-UTR was also ligated into pmirGLO construct (Promega, USA). The positive clones were then transfected into indicated cells by Lipofectamine 2000. Dual-luciferase reporter assay was performed as the previous description. Relative luciferase activity was observed by dual-luciferase reporter kit at 48 h after transfection (Promega, USA).

### 2.9. Statistical Analysis

All the data were analyzed by SPSS 15.0 software (SPSS, Inc., Chicago, IL, USA) and GraphPad Prism (version 6.0; GraphPad Software, Inc., La Jolla, CA, USA). The representative data shown as the mean ± SD were derived from experiments in triplicate. The difference that existed in the two comparison groups or multiple groups was determined by Student's *t*-test or one-way ANOVA. *P* value < 0.05 indicated an obvious difference.

## 3. Results

### 3.1. Abated circFAT1(e2) Resulted in Inhibition of Vascular Smooth Muscle Cell Viability but Induction of Cell Apoptosis

circFAT1(e2) in HUASMC and HASMC cells was silenced after transfection of si-circFAT1(e2) (Figure 1(a)). CCK-8 assay was then conducted to determine cell viability on special days. Our data revealed that reduced circFAT1(e2) greatly curbed HUASMC and HASMC cell viability (Figures 1(b) and 1(c)). To further verify reduced cell viability resulted from the aberrant cell cycle, cell apoptosis was measured by FACS after staining of Annexin V/PI. The data suggested that accumulated HUASMC and HASMC cell apoptosis was observed after downregulation of circFAT1(e2) (Figure 1(d)). Collectively, our data displayed that reduced circFAT1(e2) repressed vascular smooth muscle cell viability and promoted cell apoptosis.

### 3.2. circFAT1(e2) Sponged miR-298 and Promoted MYB Expression

Here, we wanted to validate the function of circFAT1(e2) in the progression of vascular smooth muscle. circRNAs were reported to display as ceRNAs to sponge miRNAs in tumor cells. Therefore, we searched for the probable target miRNAs, corresponding to circFAT1(e2) referred to online data. miR-298 was chosen and used in the following studies. Additionally, we deeply uncovered the downstream targets of miR-298 because miRNAs modulated the expression level of genes via targeting mRNAs. MYB was selected as one candidate for miR-298. Luciferase reporter assay was executed to confirm the above assumptions. Our data illustrated that luciferase activity could be obviously decreased in cells transfected with circFAT1(e2)-WT or MYB 3′-UTR-WT with miR-298 (Figures 2(a) and 2(b)), implying that miR-298 was a mediator between circFAT1(e2) and MYB. Collectively, our results displayed that circFAT1(e2) functioned as a sponge of miR-298, thus facilitating the expression of MYB in smooth muscle.

### 3.3. circFAT1(e2) Enhanced Vascular Smooth Muscle via miR-298/MYB Axis

Expressions of miR-298 and MYB were measured in vascular smooth muscle cell lines (HUASMC and HASMC) with si-circFAT1(e2) or miR-298, respectively. The results indicated that the silencing of circFAT1(e2) increased the expression of miR-298 (Figure 2(c)), and miR-298 had an opposite relation with MYB (Figure 2(d)). To conclude, circFAT1(e2) promoted MYB, while inhibiting miR-298 in vascular smooth muscle. Therefore, it was verified that circFAT1(e2) enhanced vascular smooth muscle via miR-298/MYB axis.

### 3.4. Detection of DEGs in Atrial Fibrillation

Next, we screened the DEGs between the normal person and patients with atrial fibrillation in GSE41177 and it was found that a total of 1982 increased genes were screened at FC > 1.5 and *P* < 0.001. As shown in Figure 3, we could observe that the gene expression patterns of the DEGs among the array data of GSE41177 were similar, demonstrating that the molecular changes were accordant and might be a novel gene marker in atrial fibrillation. Specifically, the fold change and *P* value of MYB were 1.58 and 5.48562*E* − 07, respectively. Then, the GO, KEGG, and PPI analyses of these increased genes were conducted to illustrate their potential mechanism in smooth muscle.

### 3.5. KEGG and GO Enrichment Analysis of DEGs

To delve into the biological classifications and functions of DEGs, KEGG and GO enrichment analyses were performed using DAVID.  Figure 4(a) reveals that GO terms in BP were chiefly concentrated on estrogen metabolic process (GO:0008210), positive regulation of vasoconstriction (GO:0045907), forebrain neuron differentiation (GO:0021879), endodermal cell differentiation (GO:0035987), positive regulation of protein kinase B signaling (GO:0051897), T cell differentiation (GO:0030217), regulation of vascular endothelial growth factor production (GO:0010574), positive regulation of T-helper 1 type immune response (GO:0002827), plasminogen activation (GO:0031639), and hormone secretion (GO:0046887).  Figure 4(b) shows that GO terms in CC were mainly enriched in condensed chromosome kinetochore (GO:0000777), lateral element (GO:0000800), platelet alpha granule lumen (GO:0031093), bicellular tight junction (GO:0005923), platelet alpha granule (GO:0031091), and HFE-transferrin receptor complex (GO:1990712).  Figure 4(c) demonstrates that GO terms in MF were mainly enriched in phosphatidylinositol 3-kinase activity (GO:0035004), cyclic-nucleotide phosphodiesterase activity (GO:0004112), phosphatidylinositol-4,5-bisphosphate 3-kinase activity (GO:0046934), 3′,5′-cyclic-GMP phosphodiesterase activity (GO:0047555), phosphatidylinositol bisphosphate kinase activity (GO:0052813), WW domain binding (GO:0050699), 3′,5′-cyclic-nucleotide phosphodiesterase activity (GO:0004114), cGMP binding (GO:0030553), transmitter-gated ion channel activity (GO:0022824), and ionotropic glutamate receptor activity (GO:0004970). As shown in Figure 4(d), the identified significant KEGG enrichment pathways were bladder cancer, transcriptional misregulation in cancer, nicotine addiction, one carbon pool by folate, and the p53 signaling pathway.

### 3.6. PPI Network Construction and Analysis

The PPI network of DEGs was built by STRING. Given a protein list, STRING could search for their direct interactors and then generate a PPI network composed of all these proteins and all the interactions between them. As shown in Figure 5, there were 1433 nodes and 2588 edges in the dense network, indicating that these genes were closely related to each other and together played a role in atrial fibrillation. We used the degree analysis method in Cytoscape to screen hub genes. The average degree of the identified DEGs was 3.61. The degrees of EGFR, GNG2, and FPR2 were 50, 44, and 41, respectively. We could conclude that EGFR, GNG2, and FPR2 were the most closely related to patients with atrial fibrillation.

## 4. Discussion

Smooth muscle is very common in human body tissues [17]. The abnormality of smooth muscle can trigger many diseases, like leiomyoma, bronchial asthma, and gallstones [1]. As for the treatment of smooth muscle-related diseases, there exist alarming limitations. For instance, uterine fibroids frequently belong to benign tumors of female reproductive organs, composed of smooth muscle and connective tissues [18]. Hyperuricemia promotes the occurrence of atrial fibrillation by promoting the proliferation of vascular smooth muscle [19]. Due to few symptoms of fibroids, the clinical incidence rate is much lower than the true incidence rate [20]. Currently, the main therapies, including myomectomy, intervention, and drug therapy, all have the possibility of recurrence [21].

circRNA has been reported to regulate other genes' expressions and be involved in many disease progressions. For instance, circRNA-0067835 can regulate liver fibrosis by sponging miR-155, thereby promoting FOXO3a expression [22]. Aberrant expression of hsa_cirRNA_0054633 perhaps exerts a great impact on gestational diabetes mellitus progression [23]. circFAT1(e2) is dysregulated in various diseases, including smooth muscle-related diseases [24]. It is reasonable to suppose that circFAT1(e2) plays a crucial role in smooth muscle as previously described. Therefore, we study the function and mechanism of circFAT1(e2) in vascular smooth muscle by knocking down its expression herein. Data display that reduced circFAT1(e2) represses vascular smooth muscle cell viability and promotes cell apoptosis.

circRNA is revealed to sponge miRNAs and then regulate downstream gene expression in cells [25]. Here, we screened miR-298 as the potential target of circFAT1(e2) and further regulating MYB expression level. Dual-luciferase reporter assay was performed, and the results demonstrated the luciferase activity was reduced in miR-298 overexpressed cells transfected with plasmids containing circFAT1(e2) or 3′-UTR of MYB, while no change of the luciferase activity happened in cells after transfection of mutant circFAT1(e2) or mutant 3′-UTR of MYB. Besides, low-expressed circFAT1(e2) increased miR-298 expression and overexpressed miR-298 decreased MYB in HUASMC and HASMC. Therefore, these data suggested circFAT1(e2) could sponge miR-298 and positively regulate MYB in the smooth muscle cell.

To delve into the mechanism of how circRNAs exert their functions, we investigated the downstream target of circFAT1(e2). miR-298 and MYB were found and validated to be the most potential downstream targets. Evidence has seen that the miR-298 dysregulation is associated with cancer development [26]. Arabsorkhi et al. find miR-298 has special functions in colon cancer invasion by targeting PTEN [27]. MYB belongs to a big family whose members mostly function as transcription factors via binding with DNA [23]. So far, many reports have revealed that MYB has an influence on cancers [23]. For example, Liu et al. demonstrate the value of MYB as a biomarker for adenoid cystic carcinoma prognosis [23]. In this study, based on dataset GSE41177, we found that the expression levels of MYB in 16 left atria junctions of patients with atrial fibrillation were significantly upregulated (FC = 1.58, *P* = 5.48562*E* − 07) compared with a normal person. MYB has been shown to regulate the differentiation of ESCs to VSMCs in *vitro* and plays an important role in the proliferation and hematopoiesis of VSMCs. Moreover, MYB also regulates the proliferation and differentiation of adult vessel progenitor cells that participate in neointimal remodeling.

Through the GSE41177 database, we identified 1982 DEGs in atrial fibrillation. Interestingly, 1982 DEGs were all upregulated. Then, we performed GO and KEGG analysis of these upregulated DEGs and the results indicated that they participated in many biological processes related to endodermal cell differentiation. Summing up the above discussion, it could be concluded that circFAT1(e2) facilitated the proliferation and reduced the cell apoptosis of smooth muscle via the miR-298/MYB axis. The PPI network analysis illustrated that the hub genes related to atrial fibrillation are EGFR, GNG2, and FPR2. Epidermal growth factor (EGF) is a single transmembrane domain receptor tyrosine kinase that shows the importance of growth signal transmission. Sette et al. point out that in synthetic phenotypic VSMCs, the activation of epidermal growth factor (EGF) receptor (EGFR) leads to a continuous increase in intermediate conductance. Petri et al. find that the formyl peptide receptor 2 (FPR2) has the specificity of stimulating proinflammatory and prodissociation reactions. FPR 2/ALX has a proatherosclerotic effect on bone marrow-derived cells through its influence on smooth muscle cells to promote the stability of the plaque phenotype.

In conclusion, our data reveal that miR-298 interplays with circFAT1(e2) and then affect MYB expression. circFAT1(e2) accelerates the abnormal vascular smooth muscle via sponging miR-298 and regulating MYB. circFAT1(e2)/miR-298/MYB would be considered as a new pathway to explore vascular smooth muscle development. Subsequently, MYB expression is identified to significantly upregulate in atrial fibrillation based on dataset GSE41177. And bioinformatics analysis of upregulated genes indicates that pathway endodermal cell differentiation and key genes EGFR, GNG2, and FPR2 are related to atrial fibrillation. Taken together, these findings supply a forecaster for diagnosing smooth muscle-related disease and uncover a promising strategy to treat them.

## Figures and Tables

**Figure 1:** Ablated circFAT1(e2) decreased the proliferation but induced the apoptosis of vascular smooth muscle cells. (a) Relative expression of circFAT1(e2) in HUASMC and HASMC cells transfected with si-NC (negative control) or si-circFAT1(e2). (b, c) Cellular proliferation was detected in HUASMC and HASMC cells using the CCK-8 kit at indicative time points. (d) Cellular apoptosis was demonstrated in HUASMC and HASMC cells transfected with si-NC or circFAT1(e2). ^∗^*P* < 0.05 and ^∗∗^*P* < 0.01.

**Figure 2:** circFAT1(e2) promoted MYB expression by sponging miR-298. (a, b) Luciferase reporter assay showed an interaction between miR-298 and circFAT1(e2) or MYB 3′-UTR. HASMC cells were cotransfected with luciferase reporter and miR-298 mimics. (c) circFAT1(e2) knockdown resulted in elevated expression of miR-298 in HUASMC and HASMC cells. (d) Ectopic expression of miR-298 led to decreased expression of MYB in HUASMC and HASMC cells. ^∗^*P* < 0.05 and ^∗∗^*P* < 0.01.

**Figure 3:** Hierarchical clustering diagram of the DEGs between patients with atrial fibrillation and normal person. Red represents upregulation and green represents downregulation.

**Figure 4:** GO and KEGG enrichment analysis of upregulated DEGs. (a, b, c) The identified enriched GO terms of upregulated DEGs in biological process, cellular component, and molecular function. (d) The identified enriched KEGG pathways of upregulated DEGs.

**Figure 5:** PPI network of upregulated DEGs, which is constructed by 1433 nodes and 2588 edges. Nodes refer to proteins, and edges refer to the interaction of proteins.

## Data Availability

The datasets used and/or analyzed during the current study are available from the corresponding author on reasonable request.
